The article "Factors Shaping Occupational Injustice among Resettled Syrian Refugees in the United States" was published in 2022. Journal: Occup Ther Int.

# Factors Shaping Occupational Injustice among Resettled Syrian Refugees in the United States

**DOI:** 10.1155/2022/2846896

**Published:** 2022-06-20

**Authors:** Wesam B. Darawsheh, Megan Bewernitz, Sawsan Tabbaa, Michael Justiss

**Affiliations:** ^1^Department of Occupational Therapy, School of Rehabilitation Sciences, The University of Jordan, Amman 11942, Jordan; ^2^Department of Occupational Therapy, School of Applied Health Sciences, Brooks Rehabilitation College of Healthcare Sciences, Jacksonville University, USA; ^3^School of Orthodontics, Brooks Rehabilitation College of Health Sciences, Jacksonville University, USA

## Abstract

**Background:**

There have been a limited number of studies that have focused on factors which shape the experiences of resettlement and occupational injustice among refugee populations.

**Purpose:**

To explore the factors that shape the living difficulties of Syrian refugees who were lawfully admitted into the United States and ways whereby they might interfere with shaping occupational injustice.

**Method:**

Mixed methodologies were incorporated. The living difficulty scale for refugees (LDSR) was disseminated. Semistructured interviews were conducted, and fieldnotes were collected as sources of qualitative data.

**Results:**

254 participants (mean age 36.2 ± 9.6 yrs; 159 females and 95 males) completed the survey, and nine of them participated in the semistructured interviews. Age (*p* < 0.01), region (*p* < 0.001), and time in the United States (*p* < 0.05) had significant effects on the experiences of the participants, but not gender (*p* = 0.308). Occupational injustice is an outcome of an interaction between interpersonal and contextual factors. *Practice Implications*. Occupational therapists need to assume a vital role in maximizing opportunities of engagement in meaningful occupations for Syrian refugees to counteract occupational injustice and difficulties associated with resettlement.

## 1. Introduction

Refugees are people who are forced to flee from their country of origin due to violence, oppression, or substantiated fear of persecution based on sexual orientation, gender identity, race, religion, nationality, membership in a group, or expression of certain political opinions Refugee Council United States of America [1]. Since the war in Syria in 2011, more than 5.6 million Syrians have fled from Syria to other neighboring host countries such as Jordan, Lebanon, Egypt, and Turkey to seek sanctuary The office of the United Nations High Commissioner for Refugees [2].

Resettlement is the lawful admission of vulnerable categories of people such as refugees who cannot return to their country of origin nor safely stay in host countries The office of the United Nations High Commissioner for Refugees [3]. The United States has been one of the main refugee-resettlement countries The office of the United Nations High Commissioner for Refugees [3]. Since the beginning of the 2011 fiscal year (FY) through May of the 2020 FY, there have been tens of thousands of Syrian arrivals (*n* = 21,893) to the United States, which constituted 4.2% of the total arrivals of immigrants and refugees to the United States [4].

Voluntary resettlement agencies such as the Lutheran Immigration and Refugee Services, the Church World Service, and the World Relief Corporation are responsible for the facilitation of resettling refugees in the United States [5, 6]. This is through the provision of services directed at actualizing integration of refugees in the American community, e.g., enrolment of refugees in public benefit, cultural orientation, and English as an Alternative Language (EAL) programs. The Office of Refugee Resettlement (ORR) provides funding for resettlement agencies whose practices are guided by the Refugee Act of 1980 [5, 7]. The ORR focuses on achieving expeditious economic self-sufficiency and guides resettlement agencies to push refugees toward employment upon arrival to the United States [5, 7]. However, funding and sociocultural means of support for refugees in the United States have continuously dropped since 2016, which perpetuated the nation's emphasis on early self-sufficiency and minimized the role of resettlement agencies [8–10]. Moreover, the role of resettlement agencies in the United States was deficient as evident by common experienced living and occupational difficulties among resettled refugees in the United States [11, 12].

Refugees are subjected to growing anti-immigration sentiment and structural decisions [13, 14]. For example, the decision concerning country of resettlement, per se, is dictated by the resettlement country Agbényiga et al. [15]. This in turn extenuated the feeling of powerlessness, restrained the sense of choice, and often results in experiences of separation from family members [6]. Such living difficulties interfered with the refugees' ability to perform meaningful occupations [16]. Limited accessibility to healthcare services, linguistic and social isolation, and financial and employment challenges were common occupational difficulties experienced by resettled refugees in the United States [6, 12, 14].

Indeed, there has been sufficient study that reports on the living difficulties encountered by refugees and the effect of that on hindering their adaptation and integration into the community [13, 17]. Those studies found that factors such as country of origin, level of education, socioeconomic status, time in the United States, English proficiency skills, and age impact refugees' resettlement experiences [18–20]. However, there is a scarcity of studies comparing the living experiences of refugees, in general, and Syrian refugees, in particular, across the country. Moreover, there has not been sufficient research study carried out within the field of occupational therapy or with a specific occupational science perspective.

Occupational deprivation is a common consequence of displacement [21, 22]. It is defined as a condition where an individual is unable to engage in meaningful occupations due to enforced contextual factors such as a lack of sources of sustenance, support and services, diminished safety, and separation/loss of family members [21, 23, 24]. Occupational deprivation is a form of occupational injustice, which is a state created by the contextual factors of political or economic forms [21, 23]. Occupational injustice includes other subcategories such as occupational imbalance, occupational marginalization, and occupational alienation [23]. When occupational injustice occurs, humans as occupational beings are impeded from their right to have equal opportunities to participate in meaningful occupations that meet their occupational needs and needs of self-actualization based on personal characteristics [21–24].

Forms of occupational injustice are evident in the experiences of forced migration throughout and even after resettlement [25]. Refugees are subjugated by intricate political, economic, and organizational factors that enforce occupational options and emphasize the experiences of occupational injustice [26, 27]. Opportunities for occupational participation are further minimized by limited forms of support, e.g., financial/economic, which in turn extenuates the feelings of powerlessness and loss of control and power [25, 27]. Due to that resettled-refugee populations become socially isolated, and experience exacerbated adverse psychological effects associated with perceptions of inadequacy and dependency [25, 28].

In their cross-sectional survey study of 1902 participants, Habib et al. [29] found that adult Syrian refugees in Lebanon experienced occupational deprivation in work activities. This in turn led refugee children to experience forced labor under hazardous conditions that undermined their health and led to mortality incidents and occupational deprivation from education [29]. Mirza [28] employed a grounded theoretical approach to investigate the resettlement experiences of eight Cambodian and seven Somali refugees. She found that forms of occupational injustice are to be prevalent and occupational participation is to be overlooked by American refugee policy that is preoccupied with welfare issues [28].

The literature offers a limited understanding of the eminent changes in patterns of participation and the experiences of occupational injustice associated with forced migration [21, 27]. In addition, there have been limited studies that have focused on the contextual factors that shape the experiences of resettlement and occupational injustice among refugee populations [15, 27]. Therefore, there is a need to broaden the understanding of the effects of the contextual factors shaping the experiences of occupational injustice by studying the variations in these experiences across refugee populations [21, 27]. Studies directed to fulfil this endeavor would contribute to the development of resettlement programs and to design suitable plans directed at the facilitation of refugee resettlement and adaptation [21, 27].

## 2. Aims of the Study

The experiences of Syrian refugees with resettlement, living difficulties, and occupational injustice in the United States have rarely been investigated. The aim of the current study was to explore the effects of interpersonal factors (i.e., gender, age, region of resettlement, and time in the United States) and contextual factors on shaping the living and occupational difficulties encountered by Syrian refugees who were lawfully admitted to the United States and ways whereby they might contribute to the development of occupational injustice.

## 3. Material and Methods

Ethical approval to conduct the study was granted by the institutional review board (IRB) at Jacksonville University (JU), JU IRB #2018-060.

### 3.1. Research Design

The current study was guided by the principles of the phenomenological approach. This approach allowed the generation of an in-depth knowledge concerning the unique experiences of participants [30, 31].

The study combined both qualitative and quantitative research methodologies to increase the reliability of the findings Seale et al. [32]. The design of the first stage was a nonexperimental, cross-sectional survey approach. This stage involved the dissemination of the living difficulty scale for refugees (LDSR). The second stage employed an exploratory qualitative research methodology design. Semistructured interviews were employed as a method of data collection. Fieldnotes were also used as a source of qualitative data as the triangulation of both methods for qualitative data collection increases the credibility of the findings [33].

### 3.2. Tools of Data Gathering

The LDSR was specifically developed in this study and consisted of 13 items (see Table 1 and Figure 1). Ten of its items were adapted from the Post Migration Living Difficulty Scale Silove et al. [34]. Three items were constructed based on the study conducted by Darawsheh [35] and focused on experienced difficulties associated with occupational injustice by refugees. These items were “sense of time is distorted,” “cultural differences and cultural shock,” and “my qualification is underappreciated.” Participants were asked to rate each of the 13 items on a scale of 5 ranging from “not a problem at all” to “a very serious problem.” The total score ranged between 13 and 65 where the higher scores indicate greater perception of living difficulties. The scale was developed in the English language and translated into Arabic. Both versions of the scale were reviewed by three reviewers fluent in both Arabic and English. One of them was a specialized linguist.

Preliminary analysis of data from the survey guided the development of a topic guide for the second stage of semistructured interviews. Examples of themes included in the topic guide were “the language barrier as a main living difficulty: sources and effects” and “effects of age on resettlement.” The topic guide included open-ended questions and served as pointers. Examples of the questions included were “how can age influence the experiences of resettlement?”, “What were the main challenges you encountered while living in the United States?”, and “How is it now to live in the United States compared to the beginning of your arrival? What has changed?”. Such questions were typically followed by prompts such as “Can you explain more or give an example?”. The interviews did not tackle topics of a political, criminal, or legal nature, and the designed topic guide kept the interviews on track. Researchers encouraged participants to seek professional help if they reported traumas of severe or persistent effects.

### 3.3. Participants and Procedure

In both stages, participants were required to be adult Syrian refugees (≥18 years) who had resettled in the United States following the conflict in 2011. Participants were given information about the study through invitation letters and information sheets written in both Arabic and English. Word-of-mouth was also used to illustrate the aims of the study in which the used dialogue was constructed from the invitation letter and the information sheet. The researchers read the questions and recorded answers of participants who did not possess sufficient literacy skills to participate.

The questionnaires did not require participants to disclose any private information. Participants were informed that once they submitted the questionnaires they could not withdraw their participation and that a partially or fully completed and returned questionnaire was considered as granting informed consent to participate in the survey. Concerning the interviews, all participants who agreed to participate were literate and were required to provide their written consent to participate. All of the interviewees were informed that they would be able to withdraw from the interviews at any point.

Convenience and snow-ball sampling were the main sampling methods incorporated in the study. The researchers approached participants and organizations that they could access in some states and within the limitations of time and budget. Snow-ball sampling was employed as participants in this research assisted in approaching other potential participants. Some of the members in the research team were from Arabic cultural backgrounds, which facilitated approaching potential participants. Some participants were directly approached by researchers in pocket neighborhoods allocated to Syrian refugees in Florida and New York. The researchers directly approached other participants through telephone/mobile conversations and applications, word-of-mouth, face-to-face interactions, and/or email. Some participants were also approached through closed social media groups, community centers, and organizations involved in the affairs of refugees. The personnel responsible for the social media groups, organizations, and centers were also the ones who made the first contact with participants and sent the invitation letters and information sheets.

In the first survey stage, participants were asked to voluntarily provide their contact details if they were willing to participate in the prospective semistructured interviews. Participants who provided their contact details were contacted for the second stage. In case a contacted participant changed his or her decision concerning participation, another candidate was contacted providing the allocated budget for this research allowed. The target number of interviewees was 8 to 12 and depended on reaching a point of data saturation.

Interviews were recorded and transcribed. They were conducted face-to-face as this allowed researchers to collect further data pertinent to nonverbal communications and the surrounding context. Several of the fieldnotes included critical reflections, interrelations, and interpretations which enriched the process of data analysis [36]. Arabic was the primary language of the participants and members of the research team involved in data gathering and transcription. The data were gathered and analyzed in Arabic, so there was no need for translators.

### 3.4. Data Analysis

Statistical analysis was performed using the SPSS Version 22.0 (2016, IBM Corporation, New York). Descriptive statistical analysis was employed to report on the occurrence of categorical variables. The MANOVA test was used to compare the effects of the factors of gender, age, region, and time in the United States on the items listed in the LDSR. The reliability assessment and the internal consistency reliability coefficient (Cronbach's alpha) of the LDSR were calculated. A conventional benchmark value of a Cronbach's *α* value of ≥0.7 is commonly used to indicate that most of the items measure the same construct [37]. The convergent construct validity of each item of the LDSR was calculated using the values of Pearson's correlation coefficients with the total score. For each item to be valid, Pearson's *r* was required to be more than critical value of *r*(252) = 0.162, at the 0.01 level for two-tailed test [38].

Interviews and fieldnotes were cited by the date of collection and participant's number [36]. The interpretive phenomenological analysis is a systematic and detailed approach used for analysis and was used in this study [39]. The first step involved was to get familiar with the data by reading and rereading transcripts and listening to audio recordings multiple times [40]. This procedure helped the researchers deepen their understanding of their accounts [30]. During familiarization, notes were written that served to abridge elaborative responses into short statements [40]. Further condensation of data was implemented by transforming the initial notes into concise phrases that reflected the essence of the participants' accounts [30]. Then, subthemes of conceptual similarities were grouped together under the same theme Pietkiewicz and Smith [31]. Finally, composite descriptions of the experiences of participants were written by searching for interrelations and explanations Pietkiewicz and Smith [31].

Peer debriefing was used as a measure of credibility where the process of analysis was reviewed to check for consistency in findings [41]. As participants and the main researchers involved in data gathering and analysis were speaking the same language, no language difference was presented in data gathering, transcription, and during the first stage of analyses Van Nes et al. [42]. This reduced the limitations of lost meaning associated with interpretation because the first coding phase stayed closely to the data. The second stage of analysis involved that themes, subthemes, and key quotes were subjected to peer debriefing by another two members of the research team who were native English speakers. Finally, a bilingual native English speaker revised the interpretation of the selected and presented quotes in the manuscript to ensure accurate cultural and not literal translation.

## 4. Findings

The sample consisted of 254 participants (mean age 36.2 ± 9.6 yrs): 159 females (mean age 34.4 ± 8.7 yrs) and 95 males (mean age 39.2 ± 10.2 yrs). Participants had an average time of 3.7 ± 1.3 yrs (range 1 month-7 yrs) in the United States. They lived in 13 states and three regions in the United States, i.e., Northeast, Midwest, and South. The average score of participants in the LDSR was 34.20 ± 9.27, and the score range was 50 (14-64).  Figure 2 presents the demographics of participants. Table 1 presents the scores of participants on the LDSR. Figure 1 presents the median scores of participants per item of the LDSR in descending order.

### 4.1. The Validity and Reliability of the LDSR

The results showed that items of the LDSR were characterized by high values of Cronbach's alpha (0.774), which confirmed the internal consistency of the items and the reliability of the scale. The values of Pearson's correlation coefficient with the total score for the items of the LDSR ranged between 0.344 ≤ *r* ≤ 0.671. All of which were more than the critical value for Pearson's *r*(252) = 0.162, *p* < 0.01 as shown in Table 2. All of the correlations were significant at the 0.01 level (2-tailed). These results confirmed the convergent construct validity of each item of the LDSR.

### 4.2. Findings from Interviews and Fieldnotes

Semistructured interviews were conducted with nine interviewees (mean age 40.2 ± 11.6): four females and five males. Fieldnotes were collected from the interviewees and 32 participants in the questionnaire (mean age 42.8 ± 11.5): 15 females and 17 males.  Table 3 shows the demographics of participants in the semistructured interviews and the participants who appear in the fieldnotes in Findings. Core themes and subthemes that were contemplated throughout the iterative process of analysis are presented in Figure 3.

#### 4.2.1. The Effects of Interpersonal Factors

The results of the MANOVA showed that there were significant differences in the main effects of the factors of age (*p* < 0.01), region (*p* < 0.001), and time in the United States (*p* < 0.05) but not gender (*p* = 0.308). Therefore, factors of age, region, and length of stay in the United States would contribute to the individual variations in the resettlement experiences and living and occupational difficulties experienced by participants (Table 1). The scores of the LDSR across the subgroups were evident in the findings from the interviews and fieldnotes. For example, concerning the effect of age, the youngest generation of participants helped their families to overcome the language barrier which indicated that the language barrier was more evident in older generation. This in turn hindered the older generation from pursuing their role as parents: “I feel like a fish out of water even at my own house as sometimes they [my children] talk with each other in English” (Interviewee 1, Northeast, 13 Mar 19). This also affected participants' sense of self-value and self-respect as evident in the quote by P217 (South): “I only go out with my daughter because she can speak English and translate for me . . . I feel useless like a dead duck and suppressed” (Fieldnote, 20 Feb 19).

#### 4.2.2. Contextual Factors and Systemic Barriers

Systemic barriers, such as the American refugee and allocation policies, deficient role of resettlement agencies, inefficient interpretation services, and lack of support, constituted major contextual factors and shaped the experienced living and occupational difficulties by refugees. Participants described the American refugee policy as focused on early self-sufficiency with limited means of financial support, as P220 (South) reported:

After three months, they [the resettlement agency] stopped paying the rent [from the welcome provisions]. They informed us that my husband needed to work and pay his own financial commitments. Well, how on earth was he supposed to find work with the fracture he had in his leg and without being able to speak English? (P220, South, 21 Feb 19)

This in turn extenuated the language barrier as it limited the available time for refugees to learn the English language, as P249 (South) reported: “Though I attended the classes [EAL classes], I did not learn English. Five months were not enough to learn the language. Besides, I was distracted all the time as I was worried about being late for work after” (Fieldnote, 7 Mar 19).

Participants reported that interpretation services were not consistently provided. Even when or if they were provided, such services were ineffective as reported by interviewee 4:

You cannot have interpretation services running for you all the time. . . When interpretation services are provided, they are often inefficient. For example, when you seek medical attention, you have to be precise concerning the symptoms that you or your child has. There are translators but their interpretation is often inaccurate as they often have different Arabic dialect from yours which lead to a lot of misunderstandings. Once, my daughter had constipation. I was asked [by a healthcare professional] whether she had blood coming out while she was defecating, and my answer was no… the translator mistranslated by saying that my daughter was scratching herself until blood comes out. Thus, I asked the translator to stop interpreting what I was saying. (Interviewee 4, Northeast, 13 Mar 19)

The American refugee policies and the deficient role of the resettlement agencies and organizations extenuated the experiences of separation from their families: “I have extended family members in California and I wanted to join them. The agency refused to assist us to move there and even to give us our welcome provisions, so we could manage to move by ourselves” (Interviewee 7, South, 23 Mar 19).

Thus, the contextual challenges led participants, such as P53 (Midwest) and Interviewee 6, to report that the current participation in meaningful occupations was transformed into forms of struggle experienced on a daily basis and accompanied by a feeling of despair and diminished sense of self-value: “As he struggled with a mail correspondence, P53 (Midwest) said, “We [Syrian refugees] are in underground graves because we cannot speak. When we learn the language, then we can start living our lives” (Fieldnote, 1 Feb 19).

When I used to go by bus, I used to sit by the window and pay extra attention . . . So, when my stop is nearly approaching, I could have enough time to make a gesture for the driver to stop. (Interviewee 6, South, 23 Mar 19)

#### 4.2.3. Occupational Injustice

This section shows how contextual factors interacted to shape forms of occupational injustice. Occupational deprivation was evident by the accounts of participants mainly in leisure, social, and work activities. Participants reported a feeling of discrimination and social isolation and experience occupational deprivation and marginalization from meaningful work activities as reported by P198 (Nebraska):

P198 (Midwest) had qualifications, but the language barrier hindered him from being able to utilize his certificate. This was disappointing especially when participants compared themselves to other work colleagues who had equivalent qualifications but were paid more and worked in better conditions/positions because they could speak English. (Fieldnote, 17 Feb 2019)

The allocation of participants in pocket neighborhoods was a source of deprivation from social activities: “I wished to be able to socialize more with the American citizens, but we are surrounded by neighbors who are Syrian refugees like us” (Interviewee 5, Northeast, 15 Mar 19). Experiences of deprivation from social activities were exacerbated by the separation from extended family members, which can also be attributed to the American refugee allocation policies as demonstrated in the previous section:

I miss our familiar gathering. Daily life activities that we perform with each other. I used to receive a lot of support and help in raising my children. Now my children are losing a lot as they are growing up isolated. (Interviewee 6, South, 23 March 19)

Participants reported experiences of occupational imbalance as evident by extensive engagement in work activities and deprivation from engagement in leisure activities as P247 (South) stated, “The sense of enjoyment in life is not for us, it is for our children. For us [the adults], we are struggling to make ends meet, we have no time for enjoyment” (Fieldnote, 7 March 19). Such a situation was imposed by the context and reflected a limitation in the financial capacity and support as P239 (South) reported: “Instead of spending money on leisure activities, it is more important to save that money to pay for the medical insurance” (Fieldnote, 6 March 19).

Participants even ended up experiencing occupational alienation as they became obliged to engage in meaningless work activities to make ends meet. As a result, they pursued jobs that did not match their field of expertise, as P192 (South) reported:

Back in Syria, P192 (South) used to have his own car paint and repair garage but could not resume his own work here in the United States… He described re-opening his own business here to be financially risky. Also, he explained that mixing paints to reach the accurate shades of colors requested by customers requires a great accuracy, and literacy in reading the labels on the buckets. (Fieldnote, 7 Mar 19)

## 5. Discussion

This study showed that contextual factors (i.e., levels of support, role of resettlement agencies, and American refugee policies) interacted with interpersonal factors (i.e., age, time in the United States, and region of resettlement) to shape the living difficulties, occupational injustice, and resettlement of Syrian refugees [5, 14–16, 43].

### 5.1. Effects of Interpersonal Factors

In this study, gender had insignificant effect on the experiences of Syrian refugees in the United States. This result agrees with the result of Hadley and Patil [19] who found that gender had no effect on the perceived discrimination among refugees from different countries of origins (i.e., East Africa, West Africa, and Eastern Europe) who had resettled in the United States. However, in a study conducted in the United States with Bhutanese refugees, Vonnahme et al. [44] found that female participants reported more depression symptoms compared to male participants. Therefore, the results concerning the effect of gender on the living difficulties and resettlement experiences of refuges remain controversial. This might reflect that gender is not a main determinant in shaping the experiences of resettled refugees in the United States and its effect is dependent on the interaction with other factors such as age and country of origin.

The presence of significant differences related to the region of resettlement in this study suggests the presence of disparity in the conditions and the level of services and support provided for Syrian refugees. Similar to our findings, Mirza et al. [45] also found that there are barriers related to accessibility to healthcare services among refugees in the Midwestern regions. Yun et al. [46] conducted a study among refugees in the Northeast. They found that though chronic noncommunicable conditions are prevalent among adult refugees, healthcare services were efficient in accommodating the screening and treatment needs of refugees with these conditions, supporting our findings where participants in the northeast had less difficulties with accessing healthcare services.

Several studies supported findings from this study by also showing that the time spent in the resettlement context affects the refugees' resettlement experiences. Findings from this study further our knowledge by showing that the challenges shifted from general discrimination at the beginning of their arrival (≤1 year), to issues related to work (>1-2 years), and underappreciation (≥4 years) that may affect their sense of value. These results may mirror the results of Hadley and Patil [19], who found that refugees' time in the United States was negatively associated with the experiences of discrimination, i.e., those who stay longer experience less discrimination as shown in Table 1.

Syrian refugees experienced a state of occupational imbalance evidenced by working for prolonged working hours to make ends meet. This was accompanied by experiences of occupational deprivation from leisure activities and limited the time available for refugees to acquire language proficiency skills [23]. The older age subgroups were more likely to report a language barrier as a difficulty compared to the young age subgroup (18-24 yrs), which might also reflect that they were more exposed to experience forms of occupational injustice. The language barrier created a gap in communication between the generations of refugees and negatively affected the social ties and the pattern of performance of activities such as child rearing [14].

### 5.2. Contextual Factors and Occupational Injustice

Occupational injustice was mainly evident in work, leisure, and social activities. This finding resonated with the findings of the study conducted by Rahapsari and Hill [12], who found that difficulties faced by Burmese refugees were related to employment and discrimination in the United States. Minor and Cameo [9] found a discrepancy in the percentages of employment between refugees and native-born citizens who had higher percentages of employment that affected refugees' self-sufficiency. This might reflect the presence of occupational marginalization as work opportunities and choices are limited for refugees [21, 23].

The experiences of occupational injustice become exacerbated by the language barrier, limitations in social support, and financial insufficiency [9]. Darawsheh et al. [47] conducted a follow-up study to the current investigation that focused on exploring the level and sources of support provided for fourteen resettled Syrian refugees in the United States. Darawsheh et al. [47] showed that the lack of support offered for resettled Syrian refugees to be a main shaper of their resettlement experiences and a main source of their experienced living difficulties. The lack of support was evident by the deficiency of the cultural orientation and English as a Second Language (ESL) programs and other means of provision of psychological support/treatment. The provision of interpretation services for refugees in the United States is mandatory as part of the refugee social services program [8]. However, as the literature and the participants showed, interpretation services are not efficient in addressing the needs of refugees [48]. Accordingly, participants experienced limitations in accessibility to community and healthcare services, and participation in social activities which mirrored the findings found in several studies (e.g., [14, 49]). In a center for refugees in Canada, El-Bialy and Mulay [16] reported that limited resources and means of self-sufficiently impeded refugees from performing outdoor activities, such as fishing and hiking, that could have facilitated coping/adaption and promoted integration [16]. Similarly, Hauck et al. [11] found that refugees from Burma, Bhutan, and Iraq experienced difficulties in employment and accessibility to education and healthcare services in the United States because of the language barrier. This in turn undermined refugees' sense of occupational choice and control over their own lives [14].

The United States refugee allocation of Syrian refugees together in specific pocket neighborhoods prevented the integration of Syrian refugees within the American community [13, 14, 47]. The American refugee resettlement policy is derived from the Refugee Act of 1980 (United States Public Law 96-212, 1980) [61]. Though the Act stipulates measures to reunite a refugee with a “spouse or a child” as section 207(c)(2) shows, it overlooks sociocultural and familial needs of refugees to be reunited with extended family members [7, 47]. This in turn exacerbated Syrian refugees' experiences of separation from their extended family members and deprivation from meaningful sociocultural activities [47]. In addition, recent United States' refugee policies legalized the travel bans for visitors and immigrants from Syria, pausing the resettlement procedures, and suspension of admission of Syrian refugees served as examples of contextual factors that prevented the reunion of family members and perpetuated the experiences of separation from family in the United States [50].

The American policy for refugees focuses on refugees' early economic self-sufficiency, i.e., expeditious employment upon arrival [5, 7, 47]. This policy has been implemented with a lack of sociocultural and psychosocial support, which in turn maximized the dependency of refugees on public benefits, limited their social inclusion in the society, and adversely affected their psychological status [7, 15, 47]. Thus, refugees end up experiencing occupational alienation as they become obliged to assume meaningless jobs with minimal requirements of English, low wages, and prolonged hours [6, 12, 23, 51].

### 5.3. Implications of the Study

Refugees need to acquire the know-how concerning the pattern of living, system, and regulations of the United States and the skills required to pursue meaningful work [6, 43, 47]. Refugees also need training for skills required to attain well-paid jobs to prevent their dependency on public benefits Darawsheh et al. [47]. Working with refugees is a nascent area of field of occupational therapy [52]. Regardless, occupational therapists have an integral role in offering support as their focus on enablement of meaningful occupation is associated with an imminent uplift in the sense of motivation and meaning in life [21, 35, 53]. The educational programs of occupational therapy need to integrate fieldwork experiences and training on working with refugees [47, 52, 54]. Occupational therapists need to act as advocates in accessing public services [55], which implies that part of occupational therapists' role is to navigate and maximize opportunities of engagement in meaningful work. Occupational therapists need also to act coaches and teachers of the skills and knowledge required to perform daily life activities in the United States [56].

Several studies, such as Siddiqui et al. [57] and Werge-Olsen and Vik [58] emphasized the role of occupational therapists in identifying the occupational history of refugees and employing the refugees' cultural familiarity with certain occupations to overcome the language barrier. Activity-based social training programs with a low demand on language proficiency should be offered for refugees to promote their social inclusion [47, 57, 59]. Occupational therapists need to develop and deliver training programs on living skills that are based on partnership with the refugees and the resettlement agencies and organizations [21, 35, 47, 53, 54, 57]. The involvement of the refugees is essential to steer the services offered into addressing the unique sociocultural needs of each resettled refugee population [21, 35, 47, 53, 60].

## 6. Conclusion

Contextual factors (e.g., the American refugee and allocation policies, deficient role of resettlement agencies, inefficient interpretation services, and lack of support) interact with interpersonal factors (e.g., region of resettlement, age, and time in the United States) to shape the experiences of occupational injustice among resettled Syrian refugees in the United States. Occupational therapists need to assume the role of advocates, teachers, and facilitators of participation in meaningful occupations for refugees. Future research studies need to explore the sources of experiences of occupational injustice and factors that influence the variations in these experiences. Further comparative research studies need to investigate the effects of factors such as age, country of origin, and status (i.e., citizenship and immigration) on the experiences of occupational injustice and resettlement.

## Figures and Tables

**Figure 1:** Median of scores of items of the LDSR in a descending order. (1) Not a problem at all, (2) mild problem, (3) problem, (4) serious problem, and (5) very serious problem.

**Figure 2:** Numbers and percentages of participants as arranged by subgroups.

**Figure 3:** The code system contemplated throughout the IPA. Core themes are bolded.

**Table 1:** Means and standard deviation (mean ± SD) of the LDSR scores by subgroups.

	(1)	(2)	(3)	(4)	(5)	(6)	(7)	(8)	(9)	(10)	(11)	(12)	(13)
Gender													
F	4.0 ± 1.3	2.4 ± 1.3	2.5 ± 1.4	1.8 ± 1.1	1.8 ± 1.2	2.4 ± 1.5	1.9 ± 1.3	2.0 ± 1.3	2.6 ± 1.2	3.3 ± 1.5	2.5 ± 1.3	3.1 ± 1.7	4.1 ± 1.4
M	3.9 ± 1.4	2.2 ± 1.4	2.2 ± 1.4	1.5 ± 0.8	1.7 ± 1.2	2.9 ± 1.6	2.0 ± 1.4	2.1 ± 1.4	2.5 ± 1.3	3.4 ± 1.7	2.4 ± 1.4	3.2 ± 1.8	3.9 ± 1.5
Age													
18-24 yrs	2.5 ± 1.5	2.0 ± 1.0	2.1 ± 1.1	2.1 ± 1.4	2.1 ± 1.4	2.4 ± 1.4	1.9 ± 1.3	1.8 ± 1.2	2.2 ± 1.2	3.0 ± 1.7	2.6 ± 1.4	2.7 ± 1.7	3.2 ± 1.7
25-34 yrs	4.2 ± 1.1	2.4 ± 1.2	2.3 ± 1.3	1.7 ± 0.9	1.7 ± 1.0	2.6 ± 1.5	1.8 ± 1.2	2.0 ± 1.3	2.5 ± 1.2	3.3 ± 1.5	2.4 ± 1.2	3.2 ± 1.7	4.2 ± 1.2
35-44 yrs	4.1 ± 1.3	2.5 ± 1.4	2.6 ± 1.5	1.6 ± 1.0	1.9 ± 1.3	2.6 ± 1.5	2.0 ± 1.3	2.2 ± 1.4	2.6 ± 1.3	3.4 ± 1.6	2.5 ± 1.4	3.1 ± 1.7	4.1 ± 1.3
≥45 yrs	4.1 ± 1.3	2.0 ± 1.5	2.4 ± 1.4	1.6 ± 1.0	1.6 ± 1.2	2.6 ± 1.7	2.0 ± 1.4	2.1 ± 1.5	2.7 ± 1.3	3.7 ± 1.7	2.4 ± 1.5	3.3 ± 1.8	3.9 ± 1.5
Region													
Northeast	3.7 ± 1.4	2.8 ± 1.2	2.5 ± 1.1	2.1 ± 1.1	2.2 ± 1.2	2.8 ± 1.3	2.1 ± 1.2	2.4 ± 1.2	2.1 ± 1.0	2.4 ± 1.4	2.4 ± 1.1	3.0 ± 1.5	3.6 ± 1.5
Midwest	4.3±1.2	1.8±1.2	2.5±1.5	1.3±0.5	1.4±0.9	2.3±1.6	1.3±0.8	1.3±0.8	2.7±1.0	3.3±1.8	2.6±1.5	3.6±1.8	4.3±1.3
South	4.0 ± 1.3	2.3 ± 1.3	2.3 ± 1.4	1.6 ± 1.0	1.7 ± 1.2	2.5 ± 1.6	2.0 ± 1.4	2.1 ± 1.4	2.7 ± 1.3	3.8 ± 1.4	2.4 ± 1.4	3.1 ± 1.8	4.1 ± 1.3
Time in USA													
0-1 yrs	3.8 ± 1.5	2.5 ± 1.2	2.1 ± 1.6	2.4 ± 1.9	2.0 ± 1.4	2.0 ± 1.6	1.9 ± 1.6	1.8 ± 1.5	2.9 ± 1.7	3.4 ± 1.7	2.6 ± 1.7	3.0 ± 2.1	4.3 ± 1.4
2 yrs	4.0 ± 1.3	2.4 ± 1.4	2.3 ± 1.3	1.8 ± 1.1	2.0 ± 1.3	2.7 ± 1.5	2.1 ± 1.5	2.2 ± 1.4	2.6 ± 1.3	3.6 ± 1.5	2.5 ± 1.4	3.3 ± 1.7	4.1 ± 1.3
3 yrs	3.8 ± 1.5	2.2 ± 1.2	2.3 ± 1.4	1.5 ± 0.8	1.5 ± 0.9	2.5 ± 1.5	1.7 ± 1.1	1.9 ± 1.3	2.5 ± 1.1	3.3 ± 1.6	2.5 ± 1.2	3.0 ± 1.8	4.0 ± 1.5
≥4 yrs	4.4 ± 1.1	2.7 ± 1.4	3.2 ± 1.3	1.8 ± 1.1	2.1 ± 1.4	2.6 ± 1.3	1.9 ± 1.0	2.0 ± 1.0	2.6 ± 1.2	2.7 ± 1.4	2.0 ± 1.1	2.7 ± 1.5	3.8 ± 1.4

Note: (1) language barrier, (2) cultural differences and culture shock, (3) social segregation, (4) social injustice and discrimination, (5) my qualification is underappreciated, (6) unable to find appropriate work, (7) exploitation in work, (8) bad work conditions, (9) sense of time is distorted, (10) poor access to medical care, (11) poverty and poor help with welfare, (12) fears of being sent home, and (13) separation from family and worries about them.

**Table 2:** Convergent construct validity of the items of the LDSR.

Item	Pearson's correlation	Sig. (2-tailed)
Language barrier	.368^∗∗^	.000
Cultural differences and culture shock	.551^∗∗^	.000
Social segregation	.573^∗∗^	.000
Social injustice and discrimination	.543^∗∗^	.000
My qualification is underappreciated	.544^∗∗^	.000
Not being able to find appropriate work	.614^∗∗^	.000
Exploitation in work	.663^∗∗^	.000
Bad work conditions	.671^∗∗^	.000
Sense of time is distorted (seems longer or shorter than what it really is)	.458^∗∗^	.000
Poor access to medical care (emergency, long term, dentistry, or counseling services)	.443^∗∗^	.000
Poverty and poor help with welfare	.632^∗∗^	.000
Fears of being sent home	.432^∗∗^	.000
Separation from family and worries about them	.344^∗∗^	.000

^∗∗^Correlation is significant at the 0.01 level (2-tailed).

**Table 3:** Characteristics of participants in the semistructured interviews and fieldnotes.

Participant #	Gender	Age in years	Occupation	Health status	Region of resettlement	Years in USA
Interviewees						
Int 1	F	31	Housewife	No disease	Northeast	2
Int 2	M	39	Hotel housekeeping	No disease	Northeast	2
Int 3	M	48	Dishwasher in a restaurant	Diabetes	Northeast	3
Int 4	F	34	Housewife	No disease	Northeast	3
Int 5	M	66	Unemployed	No disease	Northeast	3
Int 6	F	29	Housewife	No disease	South	4
Int 7	M	43	Unemployed	Several physical injuries/detention	South	2
Int 8	F	31	Housewife	No disease	South	2
Int 9	M	41	Constructions	No disease	South	3
Participants included in the fieldnotes						
P53	M	52	Dairy queen	Diabetes	Midwest	3
P192	M	39	Painter of houses	Irritable bowel syndrome	South	2
P198	M	32	Packaging	No disease	Midwest	2
P217	F	40	Housewife	No disease	South	3
P220	F	30	Housewife	No disease	South	3
P239	F	66	Housewife	Surgeries in abdomen and back, diabetes	South	3
P247	M	36	Trading company	No disease	South	3
P249	M	40	Gas station	No disease	South	2

Note: F: female; M: male; Int: interviewee.

## Data Availability

The data are not publicly available due to their containing information that could compromise the privacy of research participants.
